# MiR-1270 Suppresses the Malignant Progression of Breast Cancer via Targeting MMD2

This article has been retracted.

**DOI:** 10.1155/2022/3677720

**Published:** 2022-03-19

**Authors:** Shaojun Hu, Yang Song, Yu Zhou, Yu Jiao, Song Wang

**Affiliations:** ^1^Department of Oncological Surgery, First Affiliated Hospital of Jiamusi University, Jiamusi, China; ^2^Department of Pathology, First Affiliated Hospital of Jiamusi University, Jiamusi, China; ^3^Department of Galactophore, The First Hospital of Qiqihar, Qiqihar, China; ^4^Department of Galactophore, Affiliated Qiqihar Hospital, Southern Medical University, Qiqihar, China

## Abstract

We aimed to detect the clinical significance of microRNA-1270 (miR-1270) in breast cancer (BCa) development and its potential influence on malignant phenotypes of BCa cells. The miR-1270 level in paired BCa and paracancerous tissues was detected. The Kaplan–Meier method was used for the prognosis analysis of miR-1270 in BCa. The biofunctions of miR-1270 in apoptosis and proliferation of breast cancer cells were evaluated. Downstream target of miR-1270 was predicted and confirmed. The involvement of monocyte to macrophage differentiation associated 2 (MMD2) in BCa development was finally illustrated. miR-1270 was lowly expressed in BCa tissues. Lowly expressed miR-1270 was associated with tumor staging, larger tumor size, and also worse prognostic results in patients with BCa. miR-1270 overexpression suppressed proliferation and increased apoptotic rate of BCa cells. Further exploration showed that MMD2 might be the target of miR-1270. MMD2 was upregulated in BCa tissues and negatively correlated to miR-1270 level. Importantly, MMD2 significantly neutralized the above biofunctions of miR-1270 in malignant phenotypes of BCa. Lowly expressed miR-1270 is a hallmark of poor prognosis in patients with BCa. It inhibits proliferative ability and increases apoptosis in BCa by negatively regulating the MMD2 level.

## 1. Introduction

With the improvement of screening, diagnostic, and therapeutic strategies, clinical outcomes of breast cancer (BCa) have been largely advanced [1, 2]. However, BCa is still the number one killer affecting women's health [3]. It is reported that in 2018, 626,679 people died of BCa globally. In China, about 69,500 people die of BCa annually, and its mortality accounts for 15.0% and 6.9% in female cancer deaths and total cancer deaths, respectively [3–6]. A comprehensive understanding of the biological heterogeneity of BCa is still lacked. Differentiation level, therapeutic response, possibility of metastasis, and clinical prognosis vary a lot in BCa patients [7]. These vital factors can hardly be reflected through conventional examinations [8–10]. Individualized differences largely restrict the efficacy of current diagnosis and treatment [9–11]. It is necessary to develop novel molecular hallmarks and therapeutic targets that contribute to evaluate the development and prognosis in BCa [12, 13].

MicroRNAs (miRNAs) are important in cellular physiological processes [14–17]. The role of miRNAs in cancers has been concerned. Abnormally expressed miRNAs are involved in cancer cell behaviors, serving as potential hallmarks and therapeutic targets [18]. Owing to the specificity and stable expression, miRNAs bring a new direction in cancer treatment [19]. miR-1270 is previously discovered to be differentially expressed in ovarian cancer (OC), glioblastoma, and papillary thyroid cancer [20–22]. This current study attempted to investigate the clinical significance of miR-1270 in BCa.

## 2. Materials and Methods

### 2.1. Sample Collection

Fifty-seven patients with BCa participated in this study. This study was approved by the Ethics Committee of First Affiliated Hospital of Jiamusi University and performed after obtaining the informed consents.

### 2.2. CCK-8 Assay

Breast cancer cell lines (including MCF-7, SKBR3, and MDA-MB-231) and MCF-10A (a kind of normal mammary epithelial cells) were cultured at the concentration of 2 × 10^3^ cells per well. Cell Counting Kit-8 (CCK-8) assay was performed daily at different time points. After cell culture for 2 h, the optical density (OD) value per sample was measured via the microplate reader at 490 nm, and the cell activity curve was plotted.

### 2.3. Cell Apoptosis Detection

The cell suspension was suspended and then incubated with Annexin V-Fluorescein isothiocyanate (FITC) (1.25 *μ*L) in darkness for 15 minutes. The precipitant was then incubated with propidium iodide (10 *μ*L) in the darkness after being centrifugated. Finally, apoptosis was measured by the FACSCalibur system.

### 2.4. Quantitative Real-Time Polymerase Chain Reaction (qRT-PCR)

TRIzol was used to extract the total RNA. qRT-PCR was performed according to the previously established instructions. GAPDH and U6 served as the internal controls. The 2^−ΔΔCt^ method was used for the quantitative analysis. Primer sequences are given in Table 1.

### 2.5. Western Blotting

Total protein extracted from the cells was quantified via the bicinchoninic acid method. Protein samples with the adjusted same concentration were separated and then loaded on polyvinylidene fluoride membranes followed by being blocked with defatted milk (5%) for 2 h and subsequently incubated with primary antibodies at 4 C overnight. Thereafter, secondary antibodies were added for further incubation for 2 h followed by bands being exposed via the enhanced luminol-based chemiluminescent (ECL) kit.

### 2.6. Luciferase Reporting

miR-1270 mimics/NC mimics and MMD2-WT/MMD2-MUT were used to transfect cells in plates (24-well). 48 hours later, cells were lysed for the further measurement of the luciferase activity.

### 2.7. Statistical Analysis

GraphPad Prism and Statistical Product and Service Solutions 18.0 were employed for data analysis. The chi-square test was employed for the relationship analysis between level of miR-1270 and pathological indexes of BCa patients. Statistical significance was set as *P* < 0.05.

## 3. Results

### 3.1. MiR-1270 Was Lowly Expressed in BCa

QRT-PCR data showed lower expressed miR-1270 in cancer tissues than paracancerous ones (Figure 1(a)). In particular, lower abundance of miR-1270 was seen in BCa tissues with a larger tumor size (≥4 cm) and worse *T* stage (T3-4) (Figure 1(b)). miR-1270 was identically downregulated in BCa cell lines (Figure 1(c)). Meanwhile, BCa patients with lowly expressed miR-1270 exhibited poor prognosis via Kaplan–Meier results.

### 3.2. MiR-1270 Attenuated Proliferation and Stimulated Apoptosis

To uncover the biological functions of miR-1270, we constructed miR-1270 mimic at first. Transfection of miR-1270 mimic markedly upregulated miR-1270 in BCa cells (MCF-7 and SKBR3) (Figure 2(a)). Overexpression of miR-1270 reduced viability (Figure 2(b)) and colony number (Figure 2(c)) in BCa cells. In addition, overexpression of miR-1270 enhanced apoptotic rate in BCa cells (Figure 2(d)).

### 3.3. MiR-1270 Bound to MMD2

Bioinformatics analysis uncovered potential targeting sites between MMD2 and miR-12703′UTR (Figure 3(a)). Luciferase experiment further indicated that miR-1270 overexpression declined the luciferase activity, confirming that MMD2 was the downstream target. MMD2 protein level was significantly decreased in BCa cells overexpressing miR-1270 (Figure 3(b)). Upregulated MMD2 was negatively related with that of miR-1270 in cancer tissues (Figure 3(c)).

### 3.4. MMD2 Neutralized the Effects of miR-1270 on BCa Cell Phenotypes

Downregulated protein level of MMD2 in BCa cells overexpressing miR-1270 was upregulated by transfection of pcDNA-MMD2, indicating the effective transfection rate (Figure 4(a)). As expected, overexpression of MMD2 downregulated miR-1270 in BCa cells overexpressing miR-1270 (Figure 4(b)). Interestingly, the reduced viability in BCa cells with overexpression of miR-1270 was reversed by cooverexpression of MMD2 (Figure 4(c)). Increased apoptotic rate after overexpression of miR-1270 in BCa cells was also reversed by upregulated MMD2 (Figure 4(d)).

## 4. Discussion

The incidence of BCa is on the rise and the onset becomes younger [1–3]. The specific phenotype of BCa is a dominant factor influencing the efficacy of anticancer treatment [4–7].

MiRNAs, produced by pre-miRNAs under the assistant of Drosha and Dicer enzymes, can recognize and bind 3′UTR of corresponding mRNAs, thus mediating their expressions and functions [14, 15]. Functionally, miRNAs help to distinguish cancer phenotype or develop drug targets [15]. Dysfunctional miRNAs may ultimately influence cancer development [16–20].

Abnormally expressed miR-1270 is found in certain types of cancers [21]. Here, we detected miR-1270 level in BCa samples. miR-1270 showed to be downregulated in BCa cell lines and tissues, suggesting the involvement of miR-1270 in the malignant development of BCa. miR-1270 level was related to the metastasis and prognosis of the patients with breast cancer. Evidence also revealed that miR-1270 was able to suppress proliferative ability and stimulate apoptosis in BCa cells.

miRNAs negatively regulate target mRNAs by binding their UTR or CDS [14, 15]. The same gene may present different subtypes in different tissues, cells, or different stages of development. A single miRNA can target several miRNAs [14–16]. As a result, a complicated network is formed and thus influences life activities [23, 24]. In this study, MMD2 was verified to be the target gene of miR-1270 by luciferase assay. miR-1270 negatively regulated MMD2 level in BCa cells. Notably, MMD2 overexpression remarkably neutralized the biofunctions of miR-1270 on proliferation and apoptosis in BCa cells. Therefore, miR-1270/MMD2 axis was involved in the malignant progression of BCa, and these two genes may be utilized as potential hallmarks. There are also several limitations in the present study. The sample size enrolled in this study was not big enough to draw convincible conclusions. Though we studied the potential underlying molecular mechanism in this process, in vivo experiments should still be performed to further verify these findings. In future, we plan to establish overexpression and know-down of miR-1270 in animal BCa models to explore the deeper mechanism involved in the regulation of tumorogenesis.

## 5. Conclusions

Downregulated miR-1270 is associated with the malignant progression in BCa patients. miR-1270 suppresses proliferative ability and increases apoptosis in BCa by negatively regulating MMD2 level.

## Figures and Tables

**Figure 1:** miR-1270 markedly downregulated in BCa. (a) miR-1270 level measured in BCa tissues and paracancerous tissues. (b) miR-1270 level in BCa tissues classified by tumor size and T stage. (c) miR-1270 level in BCa cell lines. *∗P* < 0.05, *∗∗P* < 0.01, *∗∗∗P* < 0.001.

**Figure 2:** Overexpression of miR-1270 inhibited proliferative ability and stimulated apoptosis in BCa. (a) Transfection efficacy of miR-1270 mimic in MCF-7 and SKBR3 cells. (b) Cell viability in MCF-7 and SKBR3 cells measured via CCK-8. (c) Colony formation assay done in MCF-7 and SKBR3 cells. (d) Apoptosis rate in MCF-7 and SKBR3 cells transfected with NC mimic or miR-1270 mimic. *∗P* < 0.05.

**Figure 3:** MiR-1270 bound to MMD2. (a) Luciferase assay performed in SKBR3 and MCF-7 cells. (b) MMD2 protein level in MCF-7 and SKBR3 cells transfected with miR-1270 mimic detected via Western blotting. (c) MMD2 level in BCa and paracancerous tissues. *∗P* < 0.05, *∗∗∗P* < 0.001.

**Figure 4:** MMD2 neutralized the effects of miR-1270 on BCa cell phenotypes. (a) MMD2 protein level in cotransfected SKBR3 and MCF-7 cells. (b) MiR-1270 was detected in cotransfected MCF-7 and SKBR3 cell lines. (c) CCK-8 detected the cell viability in MCF-7 and SKBR3 cells. (d) Apoptosis rate in cotransfected MCF-7 and SKBR3 cells. *∗∗P* < 0.01.

**Table 1:** Primer sequences in this study.

Gene		Primer sequence
MiR-1270	Forward	5′-CTGGAGATATGGAAGAGCTGTGT-3′
	Reverse	5′-TGCAAAGAGCCACATAGAAGAT-3′
U6	Forward	5′-CTCGCTTCGGCAGCACA-3′
	Reverse	5′-AACGCTTCACGAATTTGCGT-3′
MMD2	Forward	5′-CGCACCCTGGCTGAACCTT-3′
	Reverse	5′-CCTCCCCACGAAGAAACTGC-3′
GAPDH	Forward	5′-CAAGGTCATCCATGACAACTTTG-3′
	Reverse	5′-GTCCACCACCCTGTTGCTGTAG-3′

## Data Availability

The datasets used and analyzed during the current study are available from the corresponding author upon request.
